# Potential Genes Associated with the Survival of Lung Adenocarcinoma Were Identified by Methylation

**DOI:** 10.1155/2020/7103412

**Published:** 2020-11-18

**Authors:** Ziyuan Shen, Chenlu He, Haimiao Chen, Lishun Xiao, Yingliang Jin, Shuiping Huang

**Affiliations:** ^1^Department of Epidemiology and Biostatistics, School of Public Health, Xuzhou Medical University, Xuzhou, Jiangsu 221004, China; ^2^Center for Medical Statistics and Data Analysis, School of Public Health, Xuzhou Medical University, Xuzhou, Jiangsu 221004, China

## Abstract

**Background:**

Lung adenocarcinoma (LUAD) is the most common pathological type of lung cancer. The purpose of this study is to search for genes related to the prognosis of LUAD through methylation based on a linear mixed model (LMM).

**Methods:**

Gene expression, methylation, and survival data of LUAD patients were downloaded from the TCGA database. Based on the LMM model, the GEMMA algorithm was used to screen the predictive genes related to LUAD survival. The Cox model was used to further screen the predicted genes, and then, protein-protein interaction (PPI) network was constructed. Through the software plugin Cytoscape MCODE 3.8.0, the most closely related genes in the PPI network module were selected for in-depth biological function analysis to further explore the interaction and correlation between genes.

**Results:**

We screened out 97 predictive genes from 18,834 genes and eliminated one gene associated with lung squamous cell carcinoma from previous studies, leaving 96 genes. The MCODE and the Kaplan-Meier curve analysis were used to finally identify two genes *ASB16* and *NEDD4* that are related to the prognosis of LUAD.

**Conclusions:**

The newly identified two genes associated with the prognosis of LUAD may provide a basis for the treatment of patients.

## 1. Introduction

Global cancer data show that the incidence and mortality rates of lung cancer again top the list [1]. Approximately 520,000 new cases are reported annually in men and 267,000 in women. Nearly 61% of the pathological subtypes of lung cancer are lung adenocarcinoma (LUAD), and lung cancer poses a serious threat to human health [2]. Pathologically, different types of cancer cells originate from different sites in the lung. LUAD refers to the mucus-secreting epithelial cells that originate from the smaller bronchial mucosa, so most adenocarcinomas are located in the peripheral part of the lung in a spherical mass close to the pleura. Unlike squamous cell lung cancer, LUAD is more likely to occur in women and nonsmokers [3]. However, smoking remains a major environmental risk factor for lung cancer [4]. Causes of high mortality from LUAD include the lack of sensitive and specific early biomarkers, high likelihood of drug resistance, and metastasis [5]. In recent years, some prognostic genes related to LUAD have been found, which provide an effective criterion for early molecular diagnosis of LUAD and greatly promote the treatment of patients. The survival rate of lung cancer is on the rise gradually. In China, the 5-year relative survival rate is about 40.5%. That is up about 10 percent from a decade ago. In this study, the new predictive gene screening model and bioinformatics analysis are used to identify the driver genes associated with LUAD survival and to provide an effective criterion for early molecular diagnosis of LUAD.

Traditional treatments for LUAD usually include surgery, chemotherapy, radiation therapy, and targeted therapy [6]. In the past few years, the research on LUAD has been focused on molecular targeted therapy, controlling the metastasis of LUAD cells, and identifying the target genes [7] regulated by LUAD stem cells. In previous studies, SNP was mainly used to predict gene expression, and it has a good performance in predicting gene expression. Previous studies have shown that genes associated with LUAD survival are concentrated in regions such as 5p15.33 and 15q.

Methylation was used to predict gene expression in order to obtain methylation-driven genes associated with LUAD prognosis. DNA methylation is one of the core elements of epigenetic modification and an important signal transduction tool for regulating genome function [4]. In addition, the change of methylation state is an important factor leading to tumor genesis, including the decrease of the methylation level in the whole genome and the abnormal increase of the local methylation level in the CpG island, which leads to the instability of the genome and the nonexpression of tumor suppressor genes. Therefore, methylation can provide an important basis for early diagnosis and prognosis of cancer and provide a new idea for further clinical application. TCGA is the cancer and tumor gene mapping project initiated by the United States in 2005. The purpose of the project is to study the genome changes in cancer by using genome analysis technology. A large-scale genome sequencing has been done, including more than 30 kinds of cancers. TCGA has laid a foundation for the classification and in-depth study of the molecular pathogenesis of LUAD [8].

To search for genes associated with the prognosis of LUAD, we used an open cancer genome atlas database The Cancer Genome Atlas (TCGA) to obtain genetic and epigenetic data on LUAD [9]. LMM is a multigene model because it assumes that all mutations have a nonzero effect on gene expression. We used the effective GEMMA algorithm to fit the LMM using the limited maximum likelihood method. The gene expression value was predicted by methylation, and predictive genes were screened (defined as genes with *R*^2^ ≥ 0.05) [10]. The COX model was used to further screen the predictive genes to obtain the genes related to the prognosis of LUAD and to identify the relationship between methylation drive and LUAD. Protein-protein interaction network analysis was performed on these genes to understand the role of methylation in the development and progression of LUAD. The core genes with the highest scores in the highest clusters were extracted by MCODE in Cytoscape software. GO enrichment analysis was performed on the core genes, and Kaplan-Meier curve analysis was drawn.

## 2. Methods and Materials

### 2.1. Data Processing and Analysis

Gene expression, methylation, and clinical data of LUAD were obtained from UCSC Xena (https://xenabrowser.net/). Samples soaked in formalin-fixed paraffin-embedded tissues were excluded. Quantile conversion was performed by using the qqnorm function in R software. The original gene expression data included 20,530 genes and 515 samples, and the methylation data came from 458 samples. Firstly, quality control was carried out on the gene expression data, and more than 50% of the zero expression was eliminated. DNA methylation levels in a group of 500 kb genes were then filtered by combining gene expression levels with DNA methylation levels. Combining the gene expression and methylation data according to the sample name, 18,834 genes and 450 samples were obtained.

A total of 450 samples were included in our analysis, and the clinical variables included age, gender, and annual smoking volume. For details, basic clinical information of patients with LUAD were summarized in Table 1. The missing values were replaced by the median.

### 2.2. Two-Step Identification of Genes Associated with the Prognosis of LUAD

#### 2.2.1. Predictive Genes Were Identified Using LMM

We bring the data into the linear mixed model. Let us first assume that all the markers are normalized to mean 0 and variance 1. Let *E*_*i*_ be an *n*-vector of the expression level of the *i*th gene measured on *n* individuals, *L*_*i*_ is the *n* × *p* matrix of DNA methylation. The simple linear model that relates DNA methylation to gene expression level is *E*_*i*_ = *L*_*i*_*c*_*i*_, where *c*_*i*_ is the *p*-vector effect value corresponding to the *i*th gene. The square correlation coefficient (*R*^2^) of the predicted value is used to measure the performance. The predicted gene expression values can be regarded as the potential effect of DNA methylation. The *R*^2^ ≥ 0.05 gene is thought to be methylation driven, and these genes are retained for further analysis.

#### 2.2.2. Cox Regression Analysis Identified the Prognostic Genes

The Cox regression model was used to further analyze the predictive genes screened by the linear mixed model and to explore the relationship between methylation-driven genes and the prognosis of LUAD [36]. It is still assumed that all the markers may be involved in the development of LUAD, and the effect size of each gene should follow a normal distribution:

(1) $$\begin{array}{c} h\left(t_{i}\;|\;E_{i},L_{i}\right)=h_{0}\left(t_{i}\right){{e^{E_{i}^{T}}}^{\beta +L_{i}^{T}}}^{\gamma },\gamma \sim N\left(0,\sigma^{2}\right), \end{array}$$

where *h*_0_(*t*) is the arbitrary baseline risk function corresponding to the reference level of the covariates, and *β* is the effect size of gene *i*, and *γ* = (*γ*^1^, *γ*^2^, ⋯, *γ*^*m*^) is the *m*-dimensional vector of the random effect size of DNA methylation; *σ*^2^ is the variance of DNA methylation. We used the false discovery method to adjust the *p* value results (FDR < 0.01).

### 2.3. Protein-Protein Interaction Network and Module Analysis

In order to mine the core regulatory genes, we constructed the protein interaction network by using the STRING database (version 11.0). We also implemented signaling pathways for these genes through Cytoscape software (version 3.8.0) and visualized them through CluePedia. Through the MCODE plugin of Cytoscape software, the most closely connected modules were selected from the constructed PPI network for in-depth biological function analysis [37]. The genes contained in the modules are the core genes.

### 2.4. Kaplan-Meier Curve Analysis

Kaplan-Meier curve analysis was used to analyze the correlation between core genes and survival. We used the original expression values of genes and the predicted expression values of methylation to calculate their effects on survival, respectively. The prognosis genes were screened with *p* < 0.05 as statistically significant difference.

### 2.5. Gene Set Enrichment Analysis (GSEA)

In order to analyze the biological characteristics of prognosis genes and their roles in the development of LUAD, the prognosis genes selected by Kaplan-Meier Curve analysis were analyzed by gene set enrichment analysis. GSEA package, clusterProfiler package, and GSEA function were used in R software to obtain the enrichment results of KEGG pathway and GO pathway, respectively. The number of permutations was set to 1,000, and a falsediscoveryrate(FDR) < 0.25 was recognized as statistically significant.

## 3. Results

### 3.1. Description of Previous Studies

Before October 2019, we searched the GWAS directory with “lung cancer, lung adenocarcinoma” as the search term and conducted a systematic literature search on EBI to preliminarily understand the previous research achievements of LUAD pathogenic genes. A total of 26 articles were included, and these studies were mainly carried out in European populations. Details of the 26 articles we have included are shown in Table 2 and Figure 1, published from 2008 to 2019. A total of 314 genes were reported. The genes associated with LUAD survival were mainly located in 5p15.33, 6p21.3, 15q25, and 17q24.3. By analyzing the GO and KEGG pathways of genes related to LUAD in GWAS, the results showed that gene enrichment molecule functions were mainly identical protein binding, and the biological processes were mainly positive regulation of transcription from RNA polymerase II promoters, and the components mainly included integral component of membrane. There were altogether 22 pathways in KEGG. Several articles confirmed that genes *TP63*, *TERT*, and *CLPTM1L* were related to the prognosis of LUAD.

### 3.2. Results of Linear Mixed Model and Cox Regression Model

After placing 18,834 genes into a linear mixed model, we measured their performance by using the predicted square correlation coefficient (*R*^2^). The results showed that there were 18,495 genes with *R*^2^ greater than or equal to 0.5.  Table 3 showed information about the ten genes with a higher *R*^2^ value. A total of 114 prognostic genes were screened by Cox regression model to eliminate the nonprotein-coding genes. Finally, 97 prognostic genes were obtained. After searching on EBI, we excluded *DTNBP1*, which was linked to lung squamous cell carcinoma in previous studies [38]. In addition, we have identified a smoking-related gene, *ASB18*, which may further influence the development of lung cancer [39].

### 3.3. Protein-Protein Interaction Network and Selection of Core Genes

In this study, the protein interaction network was built by using the STRING database (version 11.0). We put 96 genes into STRING, and the species chooses to be Homo sapiens. The PPI score parameter is set at 0.400 (indicating moderate confidence). The network contains 96 nodes and37 edges, and we hide the unconnected nodes in the network. It is worth noting that there is a strong association between the genes of *ASB16*, *ASB18*, *MYLIP*, *NEDD4*, and *ZDHHC2*. The result is shown in Figure 2.

Links between genes are visualized through CluePedia, as shown in Figure 3. Through the MCODE plugin of Cytoscape 3.8.0 software (setting parameters as degreecut − off = 2, nodescore = 0.2, *k* − core = 2, and maximumdepth = 100), the most closely connected modules were selected from the constructed PPI network for in-depth biological function analysis. It was found that the genes included in the most compact modules in the cluster were *NEDD4*, *ASB18*, *MYLIP*, and *ASB16*, and the highest scoring node in the cluster was *ASB16*.

### 3.4. Kaplan-Meier Curve Analysis Results

We used Kaplan-Meier curves to describe the survival analysis of the four selected genes, and, respectively, analyzed the original gene expression data and the gene expression data predicted by methylation. The results showed that the genes of *ASB16* and *NEDD4* had a definite effect (*p* < 0.05) on the prognosis of LUAD regardless of the original value or the predictive value, while the genes of *ASB18* and *MYLIP* had no significant effect. The specific results are shown in Figure 4.

### 3.5. GSEA Results

The GSEA analysis showed that the main functions of the *ASB16* gene were covalent chromatin modification, histone methylation, and extracellular transport; the main enrichment pathways were taste transduction, DNA replication, and nucleotide excision repair. The main functions of the *NEDD4* gene were positive regulation of multiorganism process, regulation of cytoskeleton organization, and divalent inorganic cation homeostasis; the mainly enrichment pathways were MAPK signaling pathway and pathway in cancer. The most significantly enriched signaling pathways based on their NES are shown in Table 4; partial enrichment results are shown in Figure 5.

## 4. Discussion

Lung cancer, as a malignant tumor with high morbidity and mortality in the world, is not only difficult to determine the cause of the disease but also has a poor survival rate. LUAD is the most common pathological classification of lung cancer, so it is of great research value to improve the survival rate of LUAD. The previously identified genes associated with lung cancer and LUAD survival are located mainly on chromosome 6. The enrichment analysis of these genes showed that the molecular function was mainly to selectively and noncovalently interact with the same protein or protein, and the biological process was mainly a process of activating or increasing the transcription frequency, rate, or degree of RNA polymerase II promoter. The component composition mainly included the integral component of the membrane.

In recent years, studies on the survival rate of patients with LUAD have mostly focused on the prediction of genes related to prognosis, the manipulation of the immune system in the treatment of LUAD [6], the study of smoking and the occurrence of LUAD, and the use of SNP to predict the prognosis of LUAD. This study is intended to use the new model to screen the prognostic genes associated with LUAD. The resulrs showed that the two genes were associated with prognosis of LUAD and predictive genes were selected by linear mixed model and Cox regression model. Due to too many screened genes, there was excessive analysis of biological functional analysis of signaling pathways. Therefore, we use the MCODE plugin to connect many genes with a number of genes extracted and then to separate biology related analysis. Gene *NEDD4* also enriched in multiple pathways. Previous studies have found that the loci associated with LUAD are mostly located on chromosome 5, 6, 15, and 17. In this study, the genes were *ASB16* (17q21.31) and *NEDD4* (15q21.3).

The protein encoded by *ASB16* gene is a member of the protein family which contains the SOCS box-containing (ASB) and the repeated sequence of anchor proteins. They contain the repeat sequences of anchored protein and the SOCS box domains. Ankyrin repeat sequence is a kind of protein sequences widely existing in the organism of the dead body.

The *NEDD4* gene is a founding member of the HECT ubiquitin ligase *NEDD4* family, which plays a role in the protein-degrading ubiquitin proteasome system. According to a new study, the important role of the ubiquitin-proteasome system also is after it is make full use of, can metabolic toxins such as garbage, fat, and cancer cells; the human body; and metabolic energy can stimulate cell reproducing itself in order to complete the self-metabolism of the human body repair function.

In this study, we identified two prognostic genes associated with LUAD survival, and it provided a basis for improving the survival rate of LUAD. Although the gene *ASB18* has not been determined to be associated with the prognosis of LUAD, it has been shown that it is related to smoking. Smoking is an environmental risk factor for LUAD,which can be further studied.

## 5. Conclusion

Our study identified several genes that may be associated with the survival of lung adenocarcinoma, in particular two new genes (*ASB16*, *NEDD4*)) that provide evidence for the prognosis of lung adenocarcinoma, and further studies are needed to confirm our findings.

## Figures and Tables

**Figure 1:** (a) Circular Manhattan diagram of all reported SNPs in GWAS. (b) The number of reported SNPs within 1 Mb window size in GWAS. (c) The most frequently reported genes in these articles.

**Figure 2:** Results of protein-protein interaction network analysis.

**Figure 3:** Visualize links between genes. Functionally grouped network with terms as nodes linked based on their kappa score level (≥0.3).

**Figure 4:** Kaplan-Meier curve analysis results. (a, b) The combination of gene *ASB16* expression and methylation. (c, d) The combination of gene *NEDD4* expression and methylation. (e, f) The combination of gene *ASB18* expression and methylation. (g, h) The combination of gene *MYLIP* expression and methylation. pred is the gene expression predicted by methylation.

**Figure 5:** (a, b) The combination of gene *ASB16* GO and KEGG results. (c, d) The combination of gene *NEDD4* GO and KEGG results.

**Table 1:** Basic clinical information of patients with LUAD.

Clinical parameters	Number of cases
Age (years)	
>67	193
≤67	257
Sex	
Male	209
Female	241
Number-pack-years-smoked	
>37	151
≤37	299

**Table 2:** Abstracts of articles related to LUAD.

PMID	Year	*N* (case/control)	POP	Genes	Ref
18385676	2008	1,154/1,137	European	6	[11]
18385738	2008	1,989/2,625	European	5	[12]
18780872	2008	194/219	European	5	[13]
18978787	2008	5,095/5,200	European	3	[14]
18978790	2008	3,259/4,159	European	2	[15]
19654303	2009	1.952/1,438	European	4	[16]
19836008	2009	5,739/5,848	European	7	[17]
20304703	2010	328/407	European	1	[18]
20700438	2010	584/585	East Asian	2	[19]
20871597	2010	1,004/1,900	Japanese	2	[20]
20876614	2010	1,425/3,011	Korean	1	[21].
21725308	2011	2,331/3,077	Han Chinese	4	[22]
21866343	2011	426/497	Korean	3	[23]
22797724	2012	1,695/5,333	Japanese	4	[24]
22899653	2012	14.900/29,485	European	1	[25]
23143601	2012	5,510/4,544	East Asian	9	[26]
24325914	2013	2,331/3,077	Han Chinese	4	[27]
24658283	2014	2,383/3,160	Han Chinese	5	[28]
24880342	2014	11,348/15,361	European	4	[29]
25145502	2014	354	Han Chinese	1	[30]
27393504	2016	1,737/3,605	African American	6	[31]
27501781	2016	663/4,367	Japanese	6	[32]
28604730	2017	11,273/55,483	European	208	[33]
29924316	2018	775/31,563	European	18	[34]
30104567	2018	4,972/5,501	European	1	[35]
31326317	2019	27,120/27,355	Han Chinese	3	[4]

*N*: initial sample size; POP: population ethnicity.

**Table 3:** Correlation *R*^2^ values for top ten genes.

Gene	CHR	*R* ^2^	Gene	CHR	*R* ^2^
*FLJ42875*	1	0.904	*FBXL16*	16	0.917
*LOC441869*	1	0.931	*MSLN*	16	0.952
*KCNQ1*	11	0.940	*H3F3B*	17	0.923
*MUC5B*	11	0.903	*ZNF750*	17	0.918
*CBFA2T3*	16	0.904	*ADAMTSL5*	19	0.913

**Table 4:** The most significantly enriched signaling pathways.

Gene	MSigDB collection	Gene set name	NES	*p* val	FDR
*NEDD*4	c2.cp.kegg.v7.1.symbols.gmt	KEGG_FOCAL_ADHESION	2.666	0.002	0.008
		KEGG_REGULATION_OF_ACTIN_CYTOSKELETON	2.523	0.002	0.008
		KEGG_ECM_RECEPTOR_INTERACTION	2.511	0.002	0.008
	c5.bp.v7.1.symbols.gmt	GO_GRANULOCYTE_MIGRATION	2.562	0.002	0.011
		GO_DEFENSE_RESPONSE_TO_VIRUS	2.511	0.002	0.011
		GO_SUBSTRATE_ADHESION_DEPENDENT_CELL_SPREADING	2.462	0.002	0.011

*ASB16*	c2.cp.kegg.v7.1.symbols.gmt	KEGG_TASTE_TRANSDUCTION	1.701	0.002	0.088
		KEGG_ABC_TRANSPORTERS	1.605	0.006	0.088
		KEGG_LINOLEIC_ACID_METABOLISM	1.518	0.031	0.139
	c5.bp.v7.1.symbols.gmt	GO_MRNA_SPLICE_SITE_SELECTION	1.935	0.001	0.133
		GO_HISTONE_H3_K27_METHYLATION	1.893	0.001	0.133
		GO_EXTRACELLULAR_TRANSPORT	1.871	0.001	0.133

NES: normalized enrichment score; FDR: false discovery rate.

## Data Availability

The datasets analyzed during the current study are obtained from UCSC Xena (https://xenabrowser.net/).
